# miR-15a and miR-16-1 inhibit the proliferation of leukemic cells by down-regulating WT1 protein level

**DOI:** 10.1186/1756-9966-30-110

**Published:** 2011-12-01

**Authors:** Shen-meng Gao, Chong-yun Xing, Chi-qi Chen, Si-si Lin, Pei-hong Dong, Fu-jun Yu

**Affiliations:** 1 Laboratory of Internal Medicine, The First Affiliated Hospital of Wenzhou Medical College, 2 FuXue Road, Wenzhou 325000, China; 2 Department of Hematology, The First Affiliated Hospital of Wenzhou Medical College, 2 FuXue Road, Wenzhou 325000, China; 3 Department of Infection Diseases, The First Affiliated Hospital of Wenzhou Medical College, 2 FuXue Road, Wenzhou 325000, China

**Keywords:** WT1, miR-15a, miR-16-1, proliferation

## Abstract

**Background:**

miR-15a and miR-16-1(miR-15a/16-1) have been implicated as tumor suppressors in chronic lymphocytic leukemia, multiple myeloma, and acute myeloid leukemic cells. However the mechanism of inhibiting the proliferation of leukemic cells is poorly understood.

**Methods:**

K562 and HL-60 cells were transfected with pRS-15/16 or pRS-E, cell growth were measured by CCK-8 assay and direct cell count. Meanwhile WT1 protein and mRNA level were measured by Western blotting and quantitative real-time PCR.

**Results:**

In this study we found that over-expression of miR-15a/16-1 significantly inhibited K562 and HL-60 cells proliferation. Enforced expression of miR-15a/16-1 in K562 and HL-60 cells significantly reduced the protein level of WT1 but not affected the mRNA level. However enforced expression of miR-15a/16-1 can not reduce the activity of a luciferase reporter carrying the 3'-untranslated region(3'UTR) of WT1. Silencing of WT1 by specific siRNA suppressed leukemic cells proliferation resembling that of miR-15a/16-1 over-expression. Anti-miR-15a/16-1 oligonucleotides (AMO) reversed the expression of WT1 in K562 and HL-60 cells. Finally, we found a significant inverse correlation between miR-15a or miR-16-1 expression and WT1 protein levels in primary acute myeloid leukemia (AML) blasts and normal controls.

**Conclusions:**

These data suggest that miR-15a/16-1 may function as a tumor suppressor to regulate leukemic cell proliferation potentially by down-regulating the WT1 oncogene. However WT1 is not directly targeted by miR-15a/16-1 through miRNA-mRNA base pairing, therefore more study are required to understand the mechanism by which miR-15a/16-1 downregulate WT1.

## Introduction

MicroRNAs (miRNAs) are non-coding regulatory RNAs of 21 to 25 nucleotides and regulate most of basal progress such as cell proliferation, survival, apoptosis, and differentiation by triggering either translational repression or mRNA degradation[1-3]. Recently an increasing number of data have demonstrated that almost 50% of miRNAs are located at or close to fragile sites of regions. This regions are known to be amplified or deleted in human cancer[4]. miRNAs may function as tumor suppressor genes or potential oncogenes during the initiation and progression of cancer[5]. The function of some miRNAs is dependent upon the specific cell type. On one hand miR-221 and miR-222 act as oncogenes in solid tumors, on the other hand the same miRNAs function as tumor suppressors in erythroblastic leukemia cells[6]. In animals, single-stranded miRNA binds specific mRNA through sequences that are imperfectly complementary to the target mRNA, mainly to the 3' untranslated region (UTR). The bound mRNA can be degraded, resulting in decreased level of the corresponding mRNA or remains untranslated, resulting in decreased level of the corresponding protein[1,7].

The miR-15a and miR-16-1 (miR-15a/16-1) cluster reside at a genomic region of chromosome 13q14.3, which frequently was deleted or down-regulated in the majority of chronic lymphocytic leukemia (CLL), and in a subset of mantle cell lymphomas[8]. Calin *et al*. demonstrated that in MEG-01 cells enforced expression of miR-15a/16-1 inhibited cell proliferation and induce apoptosis through targeting multiple oncogenes such as Bcl-2, WNT3A, MCL1, and CCND1 in vitro and in vivo [9,10]. However the mechanism of inhibiting the proliferation of leukemic cells is still not clear.

The Wilms' tumor gene (WT1) locating at the short arm of chromosome 11 regulates the expression of different genes like transforming growth factor beta, Bcl-2, and human telomerase reverse transcriptase[11-13]. High levels of WT1 which are detected in most cases of acute myelogeous leukemia and chronic myelogeous leukemia (CML) in blast crisis are associated with a worse long-time prognosis[14]. WT1 is firstly thought to function as tumor suppressor, but the following wildly studies support that WT1 act as oncogene[15].

In this study we reported that miR-15a/16-1 were able to significantly suppress K562 and HL-60 cells proliferation through down-regulating WT1 protein level. Either down-regulation of WT1 by siRNA significantly inhibited the proliferation of leukemic cells. Thus, these data suggest that miR-15a/16-1 may function as a tumor suppressor to influence the proliferation of leukemic cells through down-regulating WT1 protein level. However, enforced expression of miR-15a/16-1 can not reduce the activity of a luciferase reporter carrying the 3'-untranslated region (3'UTR) of WT1. This result means that miR-15a/16-1 down-regulated the expression of WT1 not through miRNA-mRNA base pairing. Whether miR-15a/16-1 downregulate other genes which interact with WT1 is not decided. Therefore more study are required to shed light of the new mechanism, which will open new avenues in understanding the mechanisms of miRNA action.

## Materials and methods

### cell lines and primary leukemic cells

K562 and HL-60 cell lines were employed for the present study. All cells were cultured in RPMI 1640 supplemented with 10% fetal bovine serum (Invitrogen, Groud Island, USA) in humidified 37°C incubator with 5% CO_2_. Primary AML cells were obtained from 20 patients with AML (2 M1 5 M2, 5 M3, 2 M4, 6 M5, the First Affiliated Hospital of Wenzhou Medical College). None of these patients had received any treatment. The diagnosis was established according to French-American-British classification. All patients gave informed consent in accordance with the Declaration of Helsinki for cryopreservation and use of the samples for molecular studies.

### RNA extraction

Bone marrow mononuclear cells from normal individuals and patients with AML were aspirated by Ficoll density gradient centrifugation (GE Healthcare, Uppsala, Sweden). Total RNA from cultured cell lines and bone marrow mononuclear cells were extracted by TRIzol (Invitrogen) Following the manufacture's protocol. RNA concentrations and quality were determined with Beckman DU6400 spectrophotometer (Beckman, USA) and gel analysis.

### qPCR for miRNA and mRNA expression

Quantitative real-time polymerase chain reaction (qRT-PCR) analysis for miR-15a and miR-16-1 was performed in triplicate with the NCode™ miRNA First-strand cDNA synthesis and SYBR^® ^Green PCR Master Mix (Applied Biosystems, Foster City, CA) according to the manufacturer's instructions. U6 snRNAs was used as the internal control. The fold-change for miR-15a/16-1 expression levels was calculated using ΔC_T _and 2^-ΔΔCT^. WT1 transcript was determined by quantitative real-time PCR using specific primer sets[16] and ABL housekeeping gene was used for normalization[17]. The following primers were used respectively, WT1: (sense strand: 5'-CAG GCT GCA ATA AGA GAT ATT TTA AG CT-3', antisense strand: 5'-GAA GTC ACA CTG GTA TGG TTT CTC A-3', Taqman probe: 5'-Fam-CTT ACA GAT GCA CAG CAG GAA GCA CAC TGA-Tamra-3'), ABL: (sense strand: 5'-GAT GTA GTT GCT TGG GAC CCA-3', antisense strand: 5'-TGG AGA TAA CAC TCT AAG CAT AAC TAA AGG T-3', Taqman probe: 5'-Fam-CCA TTT TTG GTT TGG GCT TCA CAC CAT T-Tamra-3').

### Plasmids Transfection

pRETROSUPER vector expressing miR-15a/16-1 (pRS-15/16) was constructed as previously described [10,18]. The same empty plasmid (pRS-E) was served as control. Leukemic cells were transiently transfected with 1 μg/mL (final concentration) pRS-E or pRS-15/16 vector using Lipofectamine™ LTX and PLUS™ Reagents (Invitrogen) according to the manufacturer's instructions.

### Cell counting kit-8 (CCK-8) assay and trypan-blue exclusion assay

The mock or transfected K562, HL-60 and U937 cells were seeded into 96-well plates (6.0 × 10^3 ^cells/well). Cell viability was assessed by CCK-8 assay (Dojin Laboratories, Kumamoto, Japan). The absorbance at 450 nm (A450) of each well was read on a spectrophotometer. Three independent experiments were performed in quadruplicate. Alternatively, cell viability was determined by the trypan-blue exclusion assay, and growth inhibition rate was calculated according to viable cell numbers of treated cells against numbers of untransfected cells.

### siRNA and anti-miR-15a/16-1 oligonucleotide (AMO) transfection

SiRNA sequences targeting WT1 (National Center for Biotechnology Information accession number AH003034) were synthesized. siRNA-WT1: ccauaccagugugacuuca corresponds to positions 9-27 of exon 7 within the WT1 coding sequence[19]. SiRNA-WT1 and unspecific control siRNA (N.C) were obtained from Invitrogen. SiRNA-WT1 and N.C were transfected into K562 and HL-60 cells by the aid of Hiperfect transfection reagent (Qiagen, Valencia, USA). The sequences of anti-miR-15a/16-1 oligonucleotide (AMO) were designed according to the principle of sequences complementary to mature miR-15a and miR-16-1. AMO and scramble (SCR) were chemically synthesized by Qiagen. AMO and SCR (final concentration of 50 nM) were transfected into K562 and HL-60 cells mediated by Hiperfect transfection reagent (Qiagen).

### Western blotting

Bone marrow mononuclear cells from normal individuals and patients with AML were aspirated by Ficoll density gradient centrifugation (GE Healthcare). Protein extracts from cell lines, normal individuals and patient samples prepared with RIPA lysis buffer (50 mM TrisHCl, 150 mM NaCl, 0.1% SDS, 1% NP-40, 0.5% sodiumdeoxycholate, 1 mM PMSF, 100 mM leupeptin, and 2 mg/mL aprotinin, pH 8.0) were separated on an 8% SDS-polyacrylamide gel and transferred to nitrocellulose membranes. After blocking with 5% nonfat milk, the membranes were incubated with an appropriate dilution (WT1 1:2000) of the primary antibody (Abcom, Cambridge, MA, USA), followed by incubation with the horseradish peroxidase(HRP)-conjugated secondary antibody (abcom) according to manufacturer's instructions. The signals were detected by chemiluminescence phototope-HRP kit (Cell Signaling, Danvers, MA, USA) according to manufacturer's instructions. As necessary, blots were stripped and reprobed with anti-GAPDH antibody (Abcom) as an internal control. All experiments were repeated three times with the similar results. Signal intensity of proteins was normalized against GAPDH using Quantity One (Bio-Rad).

### Luciferase reporter experiments

The 3'UTR segments from the WT1 and Bcl-2 gene were amplified by PCR from cDNA and inserted into the pGL3 control vector (Promega), using the XbaΙ site immediately downstream from the stop codon of luciferase. Bcl-2 is one of known targeted gene by miR-15a/16-1[9]. The following primer set was used to generate specific fragments: Bcl-2UTRF, 5'-CTA GTC TAG AGC CTC AGG GAA CAG AAT GAT CAG-3'; Bcl-2UTRR, 5'-CTA GTC TAG AAA GCG TCC ACG TTC TTC ATT G-3'[9]. WT1UTRF, 5'-CTA GTC TAG GTA GAC CCA AAG GTC CTT AAG TT-3'; WT1UTRR, 5'-CTA GTC TAG GAT ACC GGT GCT TCT GGA A-3'. The cells were cotransfected in 24 well plate using Lipofectamine™ LTX and PLUS™ Reagents (Invitrogen) according to the manufacturer's protocol using 0.1 ug of the firefly luciferase report vector and 0.1 ug of the control vector pRL-TK (Promega, WI, USA) containing Renilla luciferase. For each well 0.5 ug pRS-15/16 or negative control pRS-E were used. Firefly and Renilla luciferase activities were measured by dual luciferase reporter assay (Promega) after transfection. Firefly luciferase activity was normalized to Renilla luciferase activity.

### Statistical Analysis

The significance of the difference between groups was determined by Student's *t*-test. A *P *value of less than .05 was considered statistically significant. Relationships between miR-15a/16-1 and WT1 expression were explored by Pearson's correlation coefficient. All statistical analyses were performed with SPSS software (version 13).

## Results

### miR-15a/16-1 suppress the proliferation of K562 and HL-60 cells

In order to explore the functional role of miR-15a/16-1 in leukemic cells, we examined the effect of miR-15a/16-1 over-expression on the proliferation of K562 and HL-60 cell lines. The cells were transfected with either pRS-15/16 or negative control plasmid (pRS-E) for 24, 48, and 72 h. The qRT-PCR analysis confirmed that the expression of miR-15a and miR-16-1 was obviously increased in cells transfected wth pRS-15/16 compared with negative control (Figure 1A and 1B). CCK-8 assay and direct cell count showed that over-expression of miR-15a/16-1 significantly inhibited the proliferation of both K562 (*P < 0.05, Figure 1C and 1D) and HL-60 cells (* *P *< 0.05, Figure 1E and 1F). In a word, our data indicate that miR-15a/16-1 may play an important role in the proliferation of leukemic cells in vitro.

**Figure 1:** **Effects of miR-15a/16-1 on the proliferation of K562 and HL-60 cells**. K562 and HL-60 cells were transfected with pRS-15/16 or pRS-E vector (negative control) for 24, 48 and 72 hours, then the relative expressions of miR-15a/16-1 were measured by qRT-PCR (A and B). CCK-8 assay (C and E) and direct cell count (D and F) were performed when K562 and HL-60 cells were transfected with pRS-15/16 or pRS-E vector at different time periods. Data are shown as mean ± SD from three independent experiments. *P < 0.05 versus negative control.

### miR-15a/16-1 reduce WT1 protein level not through targeting mRNAs according to the degree of complementarity with their 3'UTR

Calin *et al*. showed that WT1 was a target of miR-15a/16-1 in MEG-01 cells by microarray and proteomics analysis[10]. However whether WT1 was directly targeted by miR-15a/16-1 in K562 and HL-60 cells was not verified in lab. As indicated in Figure 2A, over-expression of miR-15a/16-1 in K562 and HL-60 cells obviously reduced the protein level of WT1 at 24 and 48 h after transfection with pRS-15/16 compared with normal controls, whereas the level of WT1 mRNA was not significantly affected (Figure 2B). Then we cloned the 3'UTR region of WT1 downstream of a luciferase reporter gene and corresponding negative control into K562 and HL-60 cells, but the luciferase activity of cells transfected with pRS-15/16 was not significantly decreased compared with the negative control (Figure 2C and 2D). Bcl-2 is a target of posttranscriptional repression by miR-15 and miR-16-1, which act as a positive control[9].

**Figure 2:** **miR-15a/16-1 downregulates WT1 protein level not through targeting mRNAs according to the degree of complementarity with their 3'UTR**. (A) K562 and HL-60 cells were transiently transfected with pRS-15/16 or pRS-E vector for different time periods and subjected to western analysis with the indicated antibodies. The level of GAPDH was used as a loading control. (B) K562 and HL-60 cells were transfected with pRS-15/16 or pRS-E vector for 24 and 48 hours, then the relative expression of WT1 was measured by quantitative real-time PCR. (C and D). K562 and HL-60 cells were transfected with the pGL-3 containing Bcl-2 3'UTR or WT1 3'UTR and pRS-15/16 or pRS-E for 24 hours, relative repression fold of firefly luciferase expression was standardized to Renilla luciferase, pGL-TK.

### Anti-miR-15a/16-1 oligonucleotides (AMO) reversed the expression of WT1 in K562 and HL-60 cells

In order to investigate the effect of AMO-miR-15a/16-1 on WT1 expression, we transfected AMO-miR-15a/16-1 to K562 and HL-60 cells for 24 and 48 h. miR-15a/16-1 and U6 snRNA expression was determined by quantitative real-time PCR. U6 snRNAs were used as the internal control. The fold-change for miR-15a/16-1 expression level was calculated using ΔC_T _and 2^-ΔΔCT^, as described in the Materials and methods. As indicated in Figure 3A and 3B, AMO effectively decreased the expression of miR-15a/16-1 in K562 and HL-60 cells. Meanwhile the protein level of WT1 was increased but the mRNA level of WT1 was not affected by AMO-miR-15a/16-1 at 48 hours compared with control group (SCR) in K562 and HL-60 cells (Figure 3C and 3D).

**Figure 3:** **AMO-miR-15a/16-1 reversed the expression of WT1 in K562 and HL-60 cells (A) and (B) AMO inhibited the expression of miR-15a/16-1**. K562 and HL-60 cells were incubated with AMO-miR-15a/16-1 for 24 and 48 hours, then miR-15a/16-1 and U6 snRNA expression were determined by quantitative real-time PCR. (C) and (D) K562 and HL-60 cells were incubated with AMO-miR-15a/16-1 for 48 h, then mRNA and protein level of WT1 were detected by quantitative real-time PCR and Western blotting individually. *P < 0.01 versus SCR.

### WT1 is involved in the regulation of cell proliferation by miR-15a/16-1

Because miR-15a/16-1 inhibit leukemic cells proliferation and suppress WT1 protein expression, we are interested in examining whether miR-15/16-1 play a role in the regulation of cell proliferation via WT1 regulation. To examine the functional role of WT1 in leukemic cell proliferation, we used siRNA specific for WT1. WT1 mRNA and protein levels were estimated by quantitative real-time PCR and Western blotting individually. WT1 siRNA-treated K562 and HL-60 cells showed a significant reduction of WT1 mRNA level after 24 and 48 h as compared to k562 and HL-60 control cells (Figure 4A). The down-regulation of WT1 in k562 and HL-60 achieved up to 64% and 68% respectively at 48 hours after siRNA transfection. Furthermore the reduction of mRNA using siRNA resulted in an obvious decrease of WT1 protein level after 48 h in K562 and HL-60 cell lines (Figure 4B). Finally we observed that the growth rates of k562 and HL-60 cells were significantly reduced by siRNA-WT1 compared with negative control through CCK-8 assay (Figure 4C and 4D), which resembling that of miR-15a/16-1 over-expression.

**Figure 4:** **The role of miR-15a/16-1 in the regulation of leukemic cell proliferation**. (A) and (B) K562 and HL-60 cells were incubated with 1.5 ug siRNA-WT1, 1.5 ug N.C or neither of the above for 24 and 48 hours, then the relative expression of WT1 and the corresponding WT1 protein level were separately measured by quantitative real-time PCR and Western blotting. (C) and (D) K562 and HL-60 cells treated with siRNA or N.C or neither of the above were measured by CCK-8 assay at different time periods. Data are shown as mean ± SD from three independent experiments. *P < 0.05 versus negative control.

### The levels of miR-15a/16-1 are inversely correlated with WT1 protein expression in leukemic cells

Finally we checked for the existence of a correlation between the expression levels of miR-15a or miR-16-1 by qRT-PCR and the WT1 protein levels by Western blotting in 25 AML samples and 5 normal controls. As Figure 5A indicated, whereas in two normal control cells the levels of both miRNAs were high and the WT1 protein was expressed at low levels, in six leukemic cells both miR-15a and miR-16-1 were expressed at low levels and WT1 was highly expressed. To assess the clinical relevance of these findings, we correlated WT1 protein level with miR-15a/16-1 expression in 25 AML samples and 5 normal controls. As indicated in Figure 5B and 5C, When WT1 protein levels were plotted against that of miR-15a/16-1 in each normal control and AML samples, a significant inverse correlation was found (miR-15a verse WT1 R = -0.73 *P *< 0.01; miR-16-1 verse WT1 R = -0.76 *P *< 0.01). These data indicate that miR-15a/16-1 are inversely correlated with WT1 protein level in leukemic cells.

**Figure 5:** **WT1 protein expression is inversely correlated with miR-15a or miR-16-1 expression in AML samples and normal controls**. (A) WT1 protein levels from 2 normal controls (N1 and N2) and 6 AML samples (P1-P6) were measured by Western blotting. The numbers represent the relative expression of miR-15a and miR-16-1 in the same specimens. (B) and (C) Inverse correlation between miR-15a or miR-16-1 expression and WT1 protein level in 25 primary AML samples and 5 normal controls. A statistically significant correlation between miR-15a or miR-16-1 expression and WT1 protein level was observed by Pearson's method. WT1 verse miR-15a R = -0.73 *P *< 0.01; WT1 verse miR-16-1 R = -0.76 *P *< 0.01

## Discussion

Although miRNA signatures for leukemic cell have been established, elucidation of the role of miRNAs in leukemogenesis remains in the early stage of development[20]. Calin and others presented that miR-15a/16-1 act as tumor suppressor by inhibiting the growth of tumor engraftments of leukemic cells in nude mice *in vivo*[10]. Furthermore using microarray and proteomics analysis, they found miR-15a/16-1 exerted antileukemic effect by targeting Bcl-2, WT1, and PDCD4 [10]. We used PicTar, TargetScan, and MiRanda, the most widely used algorithms for the identification of miRNA targets, to predict the target of miR-15a/16-1. To our surprise we could not find WT1 as the predicted target of miR-15a/16-1. Then we cloned the 3'UTR region of WT1 downstream of a luciferase reporter gene and corresponding negative control into K562 and HL-60 cells, but the luciferase activity of cells transfected with pRS-15/16 was not significantly decreased compared with the negative control. This data indicate miR-15a/16-1 regulate WT1 protein expression not through targeting mRNAs according to the degree of complementarity with their 3'UTR. miR-15a/16-1 might regulate gene transcription by a different mechanism than RNA-induced silencing complex mediated protein translation inhibition and/or mRNA cleavage.

Our understanding of the mechanisms by which miRNAs mediate their effects probably reflects a tip of the iceberg. Eiring *et al*. demonstrated that the interaction between miR-328 and poly(rC)-binding protein hnRNP E2 is independent of the microRNA's seed sequence[21]. They also revealed the dual ability of a microRNA to control cell fate not only through base pairing with mRNA targets but also through a decoy activity that interferes with the function of regulatory proteins[21]. miRNAs also target the 5'UTR or the coding sequence of mRNA and contribute to their down-regulation[22]. Jing *et al*. showed that AU-rich elements (AREs) mediated instability was implicated in the regulation of gene expression by miR-15a and miR-16-1[23]. Given that the interaction of miRNAs and their target genes is complicated, more research is needed to decipher the mechanisms by which miR-15a/16-1 down-regulate WT1 protein level.

miR-15a/16-1 probably regulated the expression of WT1 through an indirect effect on WT1. Several transcription factors including GATA-1 and Sp1, which bind to DNA consensus site at the proximal promoter of the WT1 gene, can regulate the expression of WT1[24,25]. We speculated whether GATA-1 and Sp1 were the targets of miR-15a/16-1. We used PicTar, TargetScan, and MiRanda to predict whether GATA-1 and Sp1 were the targets of miR-15a/16-1. However we could not find GATA-1 and Sp1 as the predicted targets of miR-15a/16-1. Meanwhile GATA-1 and Sp1 protein levels were not decreased by Western blotting after K562 cell was transfected by miR-15a/16-1 (data not shown). These data show that GATA-1 and Sp1 are not the targets of miR-15a/16-1. Considering that many transcription factors could regulate the expression of WT1, more study are required to test the possibility that WT1 was regulated by downstream targets of miR-15a/16-1.

Overexpression of WT1 is known to modulate apoptosis by upregulation of Bcl-2 gene expression[12,26]. However Hewitt *et al*. founded that WT1 could suppress the Bcl-2 promoter in transient transfection assays[27]. Murata *et al*. did not see significant changes in Bcl-2 expression in the M1 cells which induced to express WT1 (+Ex5/-KTS)[28]. These conflicting data demonstrate that the function of WT1 is cell-type specific. Depending on the cell type being investigated, WT1 can either activate Bcl-2 and function as an oncogene or suppress Bcl-2 and function as a tumor suppressor. Although Bcl-2 is a known direct target by miR-15a/16-1[9], whether miR-15a/16-1 indirectly down-regulate Bcl-2 expression through WT1 mediated down-regulation of Bcl-2 is still not proved in lab.

Depending on the cell type, WT1 had either tumor-promoting or tumor-suppressing function[29,30]. Overexpression of WT1 in human prostate cancer cells inhibited proliferation, but the expression of WT1 in leukemic cells enhanced proliferation[31,32]. Furthermore in AML and chronic myeloid leukemia (CML) patients high level of WT1 was associated with a worse long time outcome and poor event-free survival[14,33]. Yamagami *et al*. demonstrated that loss of WT1 was associated with decreased growth of the leukemic cells and rapid induction of apoptosis, when endogenous WT1 in highly expressing leukemic cell lines and primary AML samples was decreased by antisense oligonucleotides and RNA interference[34,35]. Our data showed down-regulation of WT1 by either miR-15a/16-1 over-expression and specific siRNA significantly inhibited the proliferation of leukemic cells. This data suggest that WT1 plays an important role in leukemogenesis. As WT1 is ordinary over-expressing in AML and CML patients, targeting WT1 as possible tool against leukemic cells provides a new therapeutic option for AML and CML patients[19]. The use of miR-15a/16-1 or siRNA against WT1 will have an effect in CML patients because suppressing of WT1 expression in vitro was associated with inhibition of BCR-ABL tyrosine kinase activity[36].

## Conclusion

Our data demonstrated for the first time that over-expression of miR-15a/16-1 significantly inhibited K562 and HL-60 cells proliferation through down-regulating WT1 protein level. However miR-15a/16-1 down-regulated WT1 protein level not through targeting mRNAs according to the degree of complementarity with their 3'UTR. The most important thing is to shed light on the new mechanisms by which miRNA mediated their effect, which will open new avenues for miRNA action.

## Competing interests

The authors declare that they have no competing interests.

## Authors' contributions

SMG and CYX contributed to clinical data, samples collection, CCK8, qRT-PCR and drafted manuscript. CQC carried out Western blotting. SSL carried out plasmids, siRNA, and AMO transfection. PHD carried out Luciferase reporter experiments. FJY performed the study design, statistical analysis, and manuscript writing. All authors read and approved the final manuscript.
